# Pluronic-based nano-self-assemblies of bacitracin A with a new mechanism of action for an efficient in vivo therapeutic effect against bacterial peritonitis

**DOI:** 10.1186/s12951-018-0397-3

**Published:** 2018-09-11

**Authors:** Wei Hong, Lipeng Liu, Yining Zhao, Yinghui Liu, Dexian Zhang, Mingchun Liu

**Affiliations:** Key Laboratory of Zoonosis of Liaoning Province, College of Animal Science and Veterinary Medicine, Shenyang Agricultural University, Dongling Road 120, Shenyang, 110866 Liaoning People’s Republic of China

**Keywords:** Pluronic-based Nano-BAs, Nano-BA_P85_, Tensioactive, Membranolytic effect, Efficient therapeutic effect

## Abstract

**Background:**

Although assemblies of hydrophobic-modified bacitracin A with PLGA (Nano-BA_PLGA_) have demonstrated promising antibacterial activities against both Gram-positive and Gram-negative bacteria, the desirable antibacterial potency has remained challenging due to the low solubility of Nano-BA_PLGA_. To address this tissue, a series of Pluronic copolymers (Pluronic^®^ F127, Pluronic^®^ P123 and Pluronic^®^ P85) were selected to link the N-terminus of bacitracin A to construct Pluronic-based nano-self assemblies (Nano-BA_F127_, Nano-BA_P123_ and Nano-BA_P85_).

**Results:**

Impressively, all the newly designed Pluronic-based Nano-BAs possessed higher solubility and stronger effectiveness against both Gram-positive and Gram-negative bacteria compared with Nano-BA_PLGA_, especially the modification with Pluronic^®^ P85. Surface tension measurements indicated that Nano-BA_P85_ was much more tensioactive than Nano-BA_PLGA_, which usually translated into a good membranolytic effect. Fluorescence spectroscopy and electron microscopy analyses confirmed the speculation that the cell wall/membrane might be the main action target of Nano-BA_P85_ by permeabilizing the cell membrane and damaging the membrane integrity. In vivo results further demonstrated that Nano-BA_P85_ significantly suppressed bacterial growth and prolonged survival time in the bacterial peritonitis mouse model with negligible toxicity.

**Conclusions:**

Collectively, the membrane targeting mechanism of action is entirely distinct from those of clinically used antibacterial agents. Furthermore, the new approach of construction nanoantibiotics based on the modification of commercially available antibiotics with Pluronic copolymers is demonstrated to have an efficient therapeutic effect against bacterial infection.

**Electronic supplementary material:**

The online version of this article (10.1186/s12951-018-0397-3) contains supplementary material, which is available to authorized users.

## Background

Bacitracin A (BA) is a potent narrow-spectrum antibiotic primarily against Gram-positive bacteria through disturbing bacterial cell wall synthesis by blocking the dephosphorylation of bactoprenol [1–3]. In addition, BA can also destabilize the bacterial cytoplasmic membrane and change the morphological structure as well as permeability of the cell membrane and protoplasts, resulting in the death of bacteria [4–6]. However, Gram-negative bacteria are naturally resistant to BA due to the barrier protection of the outer membrane [7]. In addition, high nephrotoxicity is another problem limiting BA application in clinics.

Structure–activity relationships revealed that the hydrophobicity of polypeptide antibiotics plays very important roles in exhibiting the strong activity against microbes [8]. Many polymeric materials, such as aliphatic acids [9, 10], palmitoyl groups [11] and cholesterol [12], have been selected for the hydrophobic modification of polypeptide antibiotics to broaden their membrane adsorption, insertion, permeabilization and disruption potency to achieve excellent antimicrobial properties. In our previous study, we examined the possibility of modification BA with poly (d,l-lactic-co-glycolic acid) (PLGA), a biodegradable and biocompatible polymer, resulting in nano-self-assemblies with greater antimicrobial activities and lower toxicity compared with their unassembled counterparts [13]. Impressively, Nano-BA_PLGA_ was not only efficient against Gram-positive bacteria but also showed a bactericidal effect on Gram-negative bacteria, and the distribution of antibacterial activity as a function of PLGA block length was skewed towards longer PLGA chains. However, a longer PLGA block reduced the solubility of Nano-BA_PLGA_, severely compromising its application.

Pluronic copolymers consisting of ethylene oxide (EO) and propylene oxide (PO) blocks arranged in a triblock structure of EO_x_-PO_y_-EO_x_ have sparked our great interest in the chemical modification of BA due to its superior water solubility and self-assembling performance over PLGA. The number of hydrophilic EO (x) and hydrophobic PO (y) units can be altered to vary the hydrophilic-lipophilic balance [14]. Pluronics are also capable of self-assembly in water as nanosized core–shell micelles above their critical micelle concentration (CMC). Generally, the PPO segment is confined in the hydrophobic micelle core in which the methyl groups are thought to interact with solubilized drug via van der Waals interactions, while two PEO blocks face out towards the aqueous media to form the micelle corona (shell), which confers water solubility through hydrogen bonding between ether oxygen and water molecules [14]. The appeal of Pluronics lies in the fine-tuning of its physicochemical properties by modifying PEO and PPO [15]. Moreover, Pluronics have demonstrated a variety of biological effects because of their interaction with the cell membrane [16–18]. The hydrophobic PPO blocks of Pluronics are considered to become immersed in hydrophobic biomembrane areas, resulting in alternations of the structure and microviscosity (“membrane fluidization”) of lipid bilayers [19, 20].

This work explored the modification of bacitracin A with Pluronics (Pluronic^®^ F127, Pluronic^®^ P85 and Pluronic^®^ P123) to construct Pluronic-based nano-self assemblies, and their antibacterial activities and biocompatibility were studied in vivo and in vitro. The Pluronic-based Nano-BAs were expected to fulfil three sequential tasks: (1) higher solubility and stronger antibacterial activity compared with Nano-BA_PLGA_; (2) precise targeting to the infected tissue, thus reducing the nephrotoxicity of bacitracin A; and (3) a unique mechanism of action. This work showed that it was possible to obtain safer and more efficient nano-self assemblies of bacitracin A modification with Pluronics, especially with Pluronic^®^ P85. Nano-BA_P85_ significantly increased the antibacterial potency and reduced toxicity manifested in the complete cure of bacterial peritonitis in a mouse model infected by *S. aureus* and *E. coli*. Moreover, Nano-BA_P85_ is targeted to its site of action by disrupting the bacterial cell wall/membrane.

## Methods

### Reagents

Bacitracin A, stannous 2-ethylhexanoate, t-butyldimethylsilanol, triphenylsilanol, *N*,*N*′-carbonyldiimidazole (CDI), Pluronic^®^ P85, Pluronic^®^ P123, Pluronic^®^F127, Triton X-100, *N*-phenyl-1-naphthylamine (NPN), *o*-nitrophenyl-β-d-galactopyranoside (ONPG), 3,3′-dipropyl thiadicarbocynine iodide (diSC_3_-5), 4-(2-hydroxyethyl) piperazine-1-ethanesulfonic acid (HEPES), phosphatidylglycerol (PG), phosphatidylethanolamine (PE) and lipopolysaccharides (rough strains) from *Escherichia coli* F583 (Rd mutant) were purchased from Sigma-Aldrich (Shanghai,China). Mueller–Hinton broth (MHB) powder, Mueller–Hinton Agar, Salmonella Shigella Agar, Maconkey Agar and Edwards Medium (Modified) were purchased form AoBoX (Beijing,China) and used to prepare the bacterial broths according to the manufacturer’s instructions. All other reagents and chemicals were of analytical or chromatographic grade and were purchased from Concord Technology (Tianjing, China).

### Bacteria

*Escherichia coli (E. coli)* ATCC 25922, *Salmonella typhimurium* (*S. typhimurium)* ATCC 13311, *Pseudomonas aeruginosa (P. aeruginosa)* ATCC 27853, *Staphylococcus aureus* (*S. aureus*) ATCC 29213, *Streptococcus pneumoniae (S. pneumoniae)* ATCC 49619 and *Tureperella pyogenes (T. pyogenes)* ATCC 19411 were purchased from the American Type Culture Collection (Manassas, VA, USA).

### Animals

Male Kunming mice (KM mice), weighing from 20 to 25 g, were used in the experiment. KM mice were supplied by the Department of Experimental Animals, Shenyang Pharmaceutical University (Shenyang, China), and were acclimated at 25 °C and 55% humidity under natural light/dark conditions. All animal experiments were carried out in accordance with guidelines evaluated and approved by the ethics committee of Shenyang Agricultural University.

### Synthesis and characterization of copolymers

All the copolymers used in this work were home-made. The details of the synthesis and characterization of BA-Pluronic^®^F127-BA, BA-Pluronic^®^ P85-BA and BA-Pluronic^®^ P123-BA are shown in Additional file 1: Additional materials.

### Preparation and characterization of Pluronic-based Nano-BAs

Nano-BA_P85_ was prepared by the thin-film hydration method. Briefly, the copolymer (BA-Pluronic^®^ P85-BA, 100 mg) was dissolved in acetonitrile (25 mL) in a round-bottomed flask. The solvent was evaporated under reduced pressure by rotary evaporation at 40 °C for 1 h to obtain a thin film. Residual acetonitrile in the film was removed under vacuum at room temperature for another 12 h. The resultant thin film was hydrated with 20 mL of PBS (pH 7.4) at 35 °C for 30 min to obtain the Nano-BA_P85_ solution. The Nano-BA_P85_ solution was then sonicated three times for 30 s with a KQ3200DB Ultrasonic Instrument at 400 W. Nano-BA_P127_ and Nano-BA_P123_ were prepared as described above with the different copolymers BA-Pluronic^®^F127-BA and BA-Pluronic^®^ P123-BA, respectively.

The hydrodynamic diameters, particle size distributions and Zeta potential of the Pluronic-based Nano-BAs were determined with a NICOMP™ 380 ZLS (Santa Barbara, USA). Each sample was filtered through a 0.45-μm disposable filter prior to measurements. Each measurement was repeated three times, and an average value was calculated. The morphologies of Pluronic-based Nano-BAs were observed using a Hitachi HT-7700 instrument operating at an acceleration voltage of 80 kV. Samples were prepared by dipping a copper grids into each respective Pluronic-based Nano-BA solution. A few minutes after deposition, the extra solution was blotted away with a strip of filter paper and stained with phosphotungstic acid aqueous solution. The water was evaporated at room temperature for 4 h before TEM observation.

### In vitro antibacterial activity assays

The minimal inhibitory concentrations (MICs) of Pluronic-based Nano-BAs (Nano-BA_F127_, Nano-BA_P85_ and Nano-BA_P123_) were determined using a modified standard micro-dilution method [21, 22]. Briefly, the initial concentration of Pluronic-based Nano-BAs was 256 μM and was serially diluted to 0.5 μM for use. One hundred microliters of bacterial suspension (10^6^ CFU/mL) from a log-phase bacterial culture was added to 96-well microtiter plates, while 100 µL of Pluronic-based Nano-BAs was also added to each well to a final volume of 200 µL. The final concentrations of the Pluronic-based Nano-BAs ranged from 0.25 to 128 μM. Inhibition of bacterial growth was determined by measuring the absorbance at 600 nm with a multifunctional microplate reader (Tecan, Austria) after an incubation of 18 h at 37 °C. The MIC was defined as the lowest concentration that completely inhibited bacterial growth. The broth with bacteria was used as the negative control, and the tests were repeated at least three times.

### Assessment of Nano-BA_P85_ adsorption by surface tension measurements

Nano-BA_P85_ adsorption at the free air/buffer interface was assessed from surface tension measurements using an Auto Surface Tensionmeter (A201, USA) based on the Wilhelmy Plate method. Aliquots of Nano-BA_P85_ and Nano-BA_PLGA_ were injected into the buffer subphase through the side arm of the measurement cell by means of a Hamilton syringe. The final concentration of the tested Nano-BAs in the subphase ranged from 0 to 1 mM. The surface tension of the solution was measured after equilibration for 24 h. Each measurement was performed at least three times.

### Transmission electron microscope (TEM) observations

Bacterial cells of *E. coli* ATCC 25922 and *S. aureus* ATCC 29213 were grown to exponential phase in MHB at 37 °C under constant shaking at 220 rpm. After centrifugation at 1000*g* for 10 min, the cell pellets were harvested, washed twice with 10 mM PBS and re-suspended to an OD_600_ of 0.2. The cells were incubated at 37 °C with Nano-BA_P85_ for 30 min, 1 h and 2 h at 1 × MICs. Polymyxin B was used as a positive control for *E. coli* ATCC 25922, while Nano-BA_PLGA_ solution was selected as the positive control for *S. aureus* ATCC 29213. The culture media with bacteria was used as the negative control. After incubation, the cells were centrifuged at 5000*g* for 5 min. The cell pellets were harvested, washed three times with PBS and subjected to fixation with 2.5% glutaraldehyde at 4 °C overnight followed by washing with PBS twice. After pre-fixation with 2.5% glutaraldehyde at 4 °C overnight, the bacteria cells were post-fixed with 2% osmium tetroxide for 70 min. After dehydration with a graded ethanol series (50%, 70%, 90% and 100%) for 8 min each, the bacterial samples were transferred to 100% ethanol, a mixture (1:1) of 100% ethanol and acetone and absolute acetone for 10 min. Then, the specimens were transferred to 1:1 mixtures of absolute acetone and epoxy resin for another 30 min and to pure epoxy resin and incubated overnight at a constant temperature. Finally, the specimens were sectioned with an ultramicrotome, stained with uranyl acetate and lead citrate, and examined using a Hitachi HT-7700 TEM.

### Interaction of Nano-BA_P85_ with peptidoglycan

The peptidoglycan (PG) content of *S. aureus* ATCC 25923 after incubation with different formulations was determined using the bacterial PG ELISA Kit. The culture media with bacteria was used as the negative control. Briefly, bacterial cells were incubated to mid-log phase in MHB, washed three times with 10 mM PBS and diluted to an OD_600_ of 0.2 in the same buffer. Subsequently, 2 mL of cell suspension was added to a quartz cuvette and mixed with 1/4 × MIC, 1/2 × MIC, and 1 × MIC Nano-BA_P85_ and 1 × MIC Nano-BA_PLGA_ at 37 °C for 1 min, 2 min, 5 min, 10 min, 20 min and 30 min. Then, the bacterial suspension was washed three times with 10 mM PBS, and 100 µL (10^7^ CFU/mL) was added to 96-well microtiter plates. The PG content was determined according to the protocols provided by the vendor using a multifunctional microplate reader (Tecan, Austria) at 450 nm.

### Interaction of Nano-BA_P85_ with LPS

#### Assessment of Nano-BA_P85_ penetration into the LPS monolayer

Formation of the LPS monolayer was conducted as previously reported [23]. A mixture of smooth LPS and Rd mutant LPS F583 (3:1 mass ratio) was selected as the LPS monolayer. Penetration of Nano-BA_P85_ into the LPS monolayer was inferred at a constant area from the change in surface pressure Δπ, which was recorded upon injection of Nano-BA_P85_ solution beneath a lipid monolayer compressed to an initial surface pressure π_i_ between 0 and 50 mN/m. The maximal monolayer initial surface pressure π_i_^max^ was deduced from the intersection of the data fitting lines and the horizontal X-axis, for which Δπ was zero. This pressure indicates the highest initial surface pressure above which the Nano-BA_5K_ is excluded from the interface [24, 25]. Penetration of Nano-BA_P85_ into the lipid LPS monolayer was also inferred at a constant surface pressure from the change in the relative surface area ΔA/A versus time, which was recorded upon injection of Nano-BA_P85_ solution beneath the LPS monolayer compressed to an initial surface pressure π_i_ of 35 mN/m. The pressure was maintained by a feedback loop that controls the barrier positions. The syringe containing the Nano-BA_P85_ solution was positioned beyond the barriers, allowing short injections at different locations beneath the preformed monolayer. The final Nano-BA_P85_ concentrations in the subphase were 0.1 or 1 μM. The results are mean values of at least three measurements.

#### LPS binding assay

The binding affinities of Nano-BA_P85_ to LPS were examined in a displacement assay using the fluorescent dye BODIPY-TR-cadaverine. Stock solutions of LPS from *E. coli* ATCC 25922 (5 mg/mL) and BODIPY-TR-cadaverine (2.5 mg/mL) were prepared and diluted in Tris buffer (pH 7.4, 50 mM) to yield final concentrations of 25 µg/mL LPS and 2.5 µg/mL BODIPY-TR-cadaverine. Nano-BA_P85_ at concentrations of 0, 1, 2, 4, 8, 16, 32, 64 and 128 μM were incubated with the LPS-BODIPY-TR-cadaverine mixture in a flat-bottom nonpyrogenic 96-well microtiter plate at 37 °C for 1 h. The changes in fluorescence (excitation wavelength: 580 nm; emission wavelength: 620 nm) were recorded using a multifunctional microplate reader (Tecan, Austria). Polymyxin B was used as a positive control.

#### Disassociation of LPS

Dynamic light scattering measurements were used to obtain information on the ability of the Nano-BA_P85_ to dissociate the LPS oligomer, and the experiment was carried out in a Zetasizer Nano ZS90 (Malvern, UK). Before starting the experiments, the Nano-BA_P85_ and buffer solutions were filtered through 0.45-μm filters. Measurements were performed after 60 min of incubation with 1 μM LPS with and without 2 μM Nano-BA_P85_. The scattering data were collected at 90º. Each measurement was repeated three times, and an average value was calculated.

### DPH labelling of bacteria

DPH was used as a probe to examine the fluidity properties of the hydrocarbon region of the cell membrane after treatment with Nano-BA_P85_ [26]. Briefly, after a 24-h incubation, *E. coli* ATCC 25922 and *S. aureus* ATCC 29213 were washed three times with PBS and incubated with 2 µM DPH labelling solution for 1 h at 37 °C. Following the initial labelling with DPH, cells were washed twice with PBS to remove extracellular DPH and resuspended in an appropriate volume of PBS. To evaluate the kinetic effects of the tested formulations (Nano-BA_P85_, Nano-BA_PLGA_ and Pluronic^®^ P85 unimers), 30 µL of the tested formulation was added to 3 mL of cell suspension. Changes in membrane microviscosity were recorded immediately and up to 90 min following the addition of the tested formulation.

### Nano-BA_P85_-induced cytoplasmic membrane disruption

#### Nano-BA_P85_-induced dye leakage assay

Two types of liposomes were prepared as follows: PG/CL with a mass ratio of 3:1 to mimic the *S. aureus* membrane, and PG/CL/PE with a mass ratio of 2:1:7 to mimic the *E. coli* membrane [27–29]. The small unilamellar vesicles (SUVs) were prepared by a modified thin-film hydration method [30]. The lipids were dissolved in 10 mL of dichloromethane and sonicated for 1 h. The solvent was removed by rotary evaporation at 45 °C for 1 h to obtain a thin film. Residual solvent remaining in the film was further evaporated under a vacuum for another 24 h at room temperature. Calcein solution was prepared by dissolving 62 mg of calcein in 1 mL of 5.0 mM HEPES buffer (pH 7.4, 100 mM). The NaOH was added in small aliquots until the calcein dissolved, yielding a dark orange solution. The resultant thin film was hydrated with calcein solution at 35 °C for 30 min to obtain a calcein-entrapped liposome solution. The calcein-entrapped liposome solution was then separated from free calcein through a Sephadex G50 column.

The calcein release assay was performed by combining 2 mL of HEPES buffer solution (pH 7.4) and 4 mL of calcein-entrapped liposomes in a beaker, with slow stirring. Membrane permeation was detected by an increase in fluorescence with an excitation wavelength of 490 nm and an emission wavelength of 520 nm, following the addition of Nano-BA_P85_. To induce 100% dye release, 10% (v/v) Triton X-100 in 20 μL of Tris–HCl (pH 7.4) was added to dissolve the vesicles. The percentage of fluorescence intensity recovery *F*_*t*_ was calculated by the following Eq. 1:

1 $$F_{t} = \left( {I_{t} - I_{0} } \right)/\left( {I_{f} - I_{0} } \right) \times 100\%$$

where *I*_0_ is the initial fluorescence intensity, *I*_*f*_ is the total fluorescence intensity with Triton X-100, and *I*_*t*_ is the fluorescence intensity observed at equilibrium after addition of Nano-BA_P85_.

#### Cytoplasmic membrane electrical potential measurement

The ability of the Nano-BA_P85_ to alter the cytoplasmic membrane electrical potential was determined using the membrane potential-sensitive dye diSC_3_-5 [21]. Briefly, *E. coli* ATCC 25922 and *S. aureus* ATCC 29213 cells in the mid-log phase in MHB were harvested by centrifugation at 1000*g* for 10 min, washed three times, and diluted to an OD_600_ of 0.05 with 5 mM HEPES buffer (pH 7.2) containing 20 mM glucose and 100 mM KCL, respectively. Subsequently, the cell suspensions were incubated with 4 µM diSC_3_-5, and the dye fluorescence intensity was monitored at 622 nm (excitation) and 670 nm (emission) at 30 s intervals. Once the maximal amount of dye had been taken up by the bacteria, Nano-BA_P85_ at a final concentration of 1 × MIC value was added to the bacterial samples, and the fluorescence intensity change due to disruption of the membrane potential gradient across the cytoplasmic membrane was determined using a multifunctional microplate reader (Tecan, Austria) from 0 to 300 s. A blank with cells and dye was used as background. Measurements were repeated at least three times.

#### Cytoplasmic membrane permeability assay

Cytoplasmic membrane (cytoplasmic membrane) permeabilization of Nano-BA_P85_ was determined by measuring the release of cytoplasmic β-galactosidase from *E. coli* and *S. aureus* cells with ONPG as the substrate, which has been previously described [21]. In brief, *E. coli* and *S. aureus* cells were grown to mid-log phase in MHB medium containing 2% lactose at 37 °C, harvested by centrifugation, washed three times and diluted to an OD_600_ of 0.05 with 10 mM PBS (pH 7.4) containing 1.5 mM ONPG. Subsequently, 2 mL of *E. coli* and *S. aureus* cells were added to a quartz cuvette and incubated with 1 × MICs of Nano-BA_P85_, Nano-BA_PLGA_ and polymyxins B at 37 °C. OD_420_ measurements recorded from 0 to 30 min every 2 min, reflecting ONPG influx into the cells, were taken as indicators of the permeability of the inner membrane.

#### In vivo anti-infective activity of Nano-BA_P85_

Approximately 6-week-old male KM mice were used for the experiments. Mice were randomly divided into 12 groups (n = 6) and intraperitoneally injected with 10^9^ colony-forming units (CFU)/mL of *E. coli* ATCC 25922, *S. aureus* ATCC 29213 and a mixture of *E. coli* ATCC 25922 and *S. aureus* ATCC 29213 in 200 μL of sterile isotonic saline [31]. One hour after inoculation, the animals were intraperitoneally injected with 200 μL of BA solution, polymyxin B, Nano-BA_P85_ or Nano-BA_PLGA_ at a dose of 30 mg/kg, 30 mg/kg, 30 mg/kg and 30 mg/kg twice a day for 3 days. On days 2, 4, and 6, 0.2 mL of ascites was aspirated from each animal, and the number of colony-forming units (CFUs) of bacteria in ascites was measured by serial dilution of the ascites. The ascites samples were placed on agar plates for 36 h at 37 °C. The number of CFUs was counted, and the results are expressed as l g CFU/mL of ascites. The survival rate of the mice was monitored for 7 days post-infection.

### Statistical analysis

All experiments were performed at least three times. Quantitative data are presented as the mean ± standard deviation (SD). Statistical comparisons were determined by analysis of variance (ANOVA) among ≥ 3 groups or Student’s *t test* between two groups. *P*-values < 0.05 and *P*-values < 0.01 were considered statistically significant.

## Results

### Characterization of the Pluronic-based Nano-BAs

The physical characterizations of the newly designed Pluronic-based Nano-BAs (Nano-BA_F127_, Nano-BA_P85_ and Nano-BA_P123_) are summarized in Table 1. The mean diameters of the Pluronic-based Nano-BAs were all less than 100 nm, with good polydispersity indexes less than 0.1. As presented in Fig. 1, the TEM images of Pluronic-based Nano-BAs showed spherical and homogenous morphology with a particle size that correlated well with those obtained by DLS. The dark region of the micellar image was probably attributed to the outer shell formed by the hydrophilic block of BA-PEO, while the bright region corresponded to the inner core formed by the hydrophobic block of PPO [32]. All of the Pluronic-based Nano-BAs exhibited a similar slightly negative surface charge at pH 7.4. We could roughly determine the dominated component on the particle surface from the negative Zeta potential data. Craig et al. has reported that the isoelectric point of bacitracin A has been found to approximate pH 6.8, thus presenting a slight negative charge in the physiological pH range from 7.0 to 7.5 [33]. Since Pluronic copolymers are all non-ionic, this negative surface charge demonstrated the presence of a BA layer on the surface of Pluronic-based Nano-BAs.

**Table 1:** The physicochemical characterization of Nano-BAs (n = 3)

Formulations	Particle size (nm)	ξ potential (mv)	PDI
Nano-BA_P123_	99.4 ± 10.5	− 4.21 ± 0.09	0.091 ± 0.003
Nano-BA_P85_	82.6 ± 11.7	− 3.02 ± 0.11	0.087 ± 0.009
Nano-BA_F127_	78.3 ± 12.3	− 3.23 ± 0.14	0.093 ± 0.006

**Fig. 1:** TEM images of Nano-BA_P123_ (**A**), Nano-BA_P85_ (**B**) and Nano-BA_F127_ (**C**)

### Antibacterial activities of Pluronic-based Nano-BAs

The antibacterial activities of the Pluronic copolymers (Pluronic^®^ P123, Pluronic^®^ P85 and Pluronic^®^ F127) and Pluronic-based Nano-BAs (Nano-BA_P123_, Nano-BA_P85_ and Nano-BA_P127_) were determined against both Gram-negative and Gram-positive bacteria. All the copolymers (Pluronic^®^ P123, Pluronic^®^ P85 and Pluronic^®^ F127) showed no visible antibacterial activities against both Gram-negative and Gram-positive bacteria, with MICs > 128 µM (data not shown). As expected (Table 2), all of the newly designed Pluronic-based Nano-BAs possessed a stronger effectiveness against both Gram-positive and Gram-negative bacteria compared with Nano-BA_PLGA_. Nano-BA_P85_ showed desirable antibacterial potential and even exhibited comparable efficiency against Gram-negative bacteria to polymyxin B. Thus, Nano-BA_P85_ was selected for future studies.

**Table 2:** Antibacterial activities of the tested formulations (MIC)

Formulations	MIC^a^ (µM)					
	Gram-positive				Gram-negative	
	*S. aureus* ATCC29213	*S. pneumoniae* ATCC49619	*A. pyogenes* ATCC19411	*E. coli* ATCC25922	*P. aeruginosa* ATCC27853	*S. typhimurium* ATCC13311
BA solution	2	4	4	> 128	> 128	> 128
Nano-BA_PLGA_	1	2	2	16	32	32
Nano-BA_F127_	0.5	1	1	8	16	16
Nano-BA_P123_	0.5	1	1	4	8	4
Nano-BA_P85_	0.5	0.5	1	1	2	2
Polymyxin B	> 128	> 128	> 128	1	1	2

^a^Minimal inhibitory concentrations (MICs) were determined as the lowest concentration of the tested copolymers that inhibited bacterial growth

### Behaviour of BA-Pluronics-BA at the air/buffer interface

The adsorption of BA-Pluronics-BA (BA-Pluronic^®^ P85-BA, BA-Pluronic^®^ P123-BA and BA-Pluronic^®^ F127-BA) and BA-PLGA_PLGA_-BA at the air/solution interface was detected by surface tension measurements. As shown in Fig. 2, for BA-Pluronic^®^ P85-BA, the surface tension of the buffer without copolymer was initially 58.28 mN/m, and at a low copolymer concentration, the surface tension decreased with increasing concentration, in accordance with Gibbs adsorption isotherm. The decrease in surface tension was due to the distribution of the BA-Pluronic^®^ P85-BA monomers to the air/water interface, indicating that the BA-Pluronic^®^ P85-BA monomers were free within this concentration. A change in slope (“a” first break) was observed at a characteristic concentration (approximately 1 × 10^−3^ g/L). Then, the surface tension values continued to decrease until a plateau was reached (“b” second break), after which the surface tension values remained approximately constant upon further increasing the concentration of BA-Pluronic^®^ P85-BA monomers up to “c”. At the break in the high-concentration region of the surface tension curve (“b”) corresponding to the CMC value (approximately 1.42 × 10^−2^ g/L), the BA-Pluronic^®^ P85-BA monomers began to form micelles (Nano-BA_P85_) due to the physical interactions between the hydrophobic blocks, leading to a reduction in the number of BA-Pluronic^®^ P85-BA monomers at the air/water interface. In contrast, the origin of the low-concentration break (“a”) was less clear and has been attributed to the formation of “monomolecular” micelles, the presence of impurities, and the arrangement of the copolymer molecules adsorbed on the air/water interface at complete surface coverage. Further increasing the concentration of BA-Pluronic^®^ P85-BA from “c” to “d” caused the surface tension to begin to decrease because Nano-BA_P85_ was saturated in the buffer and the excessive BA-Pluronic^®^ P85-BA monomers were again distributed to the air/water interface, leading to a decrease in surface tension. After the concentration increased above “d”, the surface tension remained constant due to the limited solubility of BA-Pluronic^®^ P85-BA monomers in the buffer. BA-PLGA-BA was chosen for comparison and appeared to be much less tensioactive than BA-Pluronic^®^ P85-BA. Overall, the BA-Pluronic^®^ P85-BA was highly surface active, which usually translates into a good membranolytic effect.

**Fig. 2:** Surface tension changes upon addition of BA-Pluronic^®^ P85-BA and BA-PLGA_5K_-BA at various concentrations (n = 6). Data are expressed as the mean ± standard deviation (error bars)

### Transmission electron microscopy (TEM) observation

TEM was employed to study the morphological features and intracellular alternation of bacterial cells treated with Nano-BA_P85_. The results indicated that, in comparison to the negative control (Fig. 3A) with a smooth surface and dense internal structure, Nano-BA_P85_ (Fig. 3C–E) induced a significant reduction in the integrity of the *E. coli* membrane in a time-dependent manner. After treatment with Nano-BA_P85_ (Fig. 3C) for 30 min, the *E. coli* retained their cytoplasmic membrane integrity, although a slight leakage of cellular cytoplasmic content was observed. After 2 h of treatment, the outer membrane of the *E. coli* cells appeared detached form the inner membrane, and the cells displayed the formation of vacuoles in the cytoplasm; some cells even became ghost cells with a large amount of leakage of intracellular contents (Fig. 3E). Moreover, distortion, blebbing or breakage of the cell wall treated with Nano-BA_P85_ was evident and could be observed at 1 × MIC after 2 h of treatment (Fig. 4D).

**Fig. 3:** TEM micrographs of *E. coli* ATCC 25922 treated with the Negative control (**A**) Nano-BA_PLGA_ (**B**) Nano-BA_P85_ with an incubation time of 30 min (**C**) 1 h (**D**) 2 h (**E**) and Polymyxin B (**F**)

**Fig. 4:** TEM micrographs of *S. aureus* ATCC 29213 treated with the Negative control (**A**), Nano-BA_PLGA_ (**B**), Nano-BA_P85_ with an incubation time of 30 min (**C**), 1 h (**D**), 2 h (**E**) and Polymyxin B (**F**)

### Assessment of the effect of Nano-BA_P85_ on the bacterial cell wall

PG is thought to be the major structural component of the cell wall of Gram-positive bacteria, forming a protective wall to resist a variety of host defence molecules [34]. The fluctuation of PG content after incubation with Nano-BA_P85_ was further evaluated. As shown in Fig. 5, after treatment with Nano-BA_P85_, the PG content of *S. aureus* ATCC 29213 decreased sharply in response to the change in drug concentration and incubation time. The limited PG content in the cell wall suggested a loss of completeness.

**Fig. 5:** Effects of Nano-BA_P85_ on the PG content of *S. aureus* ATCC 292139

### Interaction of Nano-BA_P85_ with LPS

#### Insertion experiments of Nano-BA_P85_ with the LPS monolayer at a constant surface area and pressure

The ability of Nano-BA_P85_ to permeabilize the LPS monolayer was first examined using surface tension measurements. In agreement with recently reported data for *E. coli* smooth strain LPS [35], we were also not able to form stable monolayers of smooth strain LPS from *E. coli*. Thus, a mixture of smooth LPS and Rd mutant LPS F583 (3:1 mass ratio) that allowed the formation of stable monolayers was selected for use in this study. The mixed LPS monolayer was considered as a relevant external leaflet model since it contained LPS in its natural form with complete mobile and flexible oligosaccharide chains immersed in the aqueous subphase. Thus, it appeared to be a relevant biomimetic model of the outer leaflet of the bacterial outer membrane to study Nano-BA_5K_ penetration.

Figure 6a shows the surface pressure increments (Δπ) with respect to the initial surface pressure of the mixed 3:1 LPS monolayer (π_i_) upon injection of Nano-BA_P85_ and Nano-BA_PLGA_ at 0.1 and 1 μM. Analysis of the adsorption-penetration curves showed evidence of dissimilar behaviours of the two agents in contact with the mixed LPS 3:1 monolayer. Nano-BA_PLGA_ had limited effect on the surface tension among the tested concentrations (0.1 and 1 μM). By contrast, the absolute values of the curve slopes were significantly higher for Nano-BA_P85_ than Nano-BA_PLGA_ for each concentration studied. The Δπ–π_i_ plot demonstrated effective penetration of Nano-BA_P85_ into the monolayer at initial surface pressures, even at low concentrations. The difference in slope between 0.1 and 1 μM was significantly pronounced due to the influence of its high surface activity on its adsorption/penetration process at concentrations higher than its CMC. In addition, at the initial pressure of 35 mN/m, the Nano-BA_PLGA_ was unable to induce increments of surface pressure, whereas the Nano-BA_P85_ could still produce a Δπ of 3.2 mN/m, which also reflected the higher affinity of Nano-BA_P85_ for the mixed LPS monolayer, especially at the 1 μM concentration. Thus, the surface pressure of 35 mN/m appeared to be a pivot value in the penetration pattern of the Nano-BA_P85_ and Nano-BA_PLGA_, and it was chosen as the initial surface pressure at which further insertion experiments were subsequently performed.

**Fig. 6:** Δπ–π_i_ relationships in constant area mode induced by the injection of Nano-BA_5K_ (0.1 μM), Nano-BA_5K_ (1 μM), Nano-BA_P85_ (0.1 μM) and Nano-BA_P85_ (1 μM) beneath the mixed LPS 3:1 monolayers (**a**). Relative surface area change (%) upon injection of Nano-BA_5K_ (0.1 μM), Nano-BA_5K_ (1 μM), Nano-BA_P85_ (0.1 μM) and Nano-BA_P85_ (1 μM) beneath the mixed LPS 3:1 monolayers (**b**). The binding affinity of Nano-BA_P85_ to LPS from *E. coli* ATCC 25922 was determined by the BODIPY-TR-cadaverine displacement method (**c**). Size distribution of LPS. (**d**) and size distribution of LPS in the presence of Nano-BA_P85_ (**e**). Representative results from six individual observations are shown as the mean ± SD in each group

Insertion experiments in constant pressure mode have been performed with the mixed LPS 3:1 monolayer compressed to the initial surface pressure of 35 mN/m to examine the contribution of hydrophobic interactions between Nano-BA_P85_ and lipid molecules. Figure 6b presents the relative area increase with respect to the time after injection of Nano-BA_P85_ and Nano-BA_PLGA_ into the subphase beneath the monolayers. The kinetics of the area increase were different for the mixed LPS 3:1 monolayer after injection of Nano-BA_P85_ with 0.1 and 1 μM, respectively. At the 0.1 μM concentration, a transient higher adsorption regime (~+ 39%) was observed 20 min after injection, before a decrease to the final value of + 21.5% was obtained 30 min after injection. A strikingly different insertion behaviour was observed for the Nano-BA_P85_ at a concentration of 1 μM. Above the CMC, at 1 μM, the relative area increase reached 70% with the mixed LPS monolayer at 20 min after the injection. After 20 min, the compression barrier reached its stop position after a full expansion, explaining the observed sudden plateau. Nano-BA_PLGA_ exhibited relatively weak penetrating ability across the mixed LPS monolayer at the tested concentrations characteristic of a limited increase in ΔA/A.

#### Binding ability of Nano-BA_P85_ to LPS

A fluorescence-based displacement assay with BODIPY-TR-cadaverine was performed to examine the binding ability of Nano-BA_P85_ to LPS. The fluorescence of BODIPY-TR-cadaverine is quenched upon binding to LPS, and the displacement of BODIPY-TR-cadaverine by Nano-BA_P85_ results in dequenching of fluorescence. Nano-BA_P85_ showed a similar dequenching effect to that observed with polymyxin B, a decapeptide antibiotic that is generally used as a Ref. [36], suggesting effective binding to LPS. In comparison to Nano-BA_P85_, Nano-BA_PLGA_ demonstrated a weaker potency for displacing BODIPY-TR-cadaverine from its binding to LPS (Fig. 6c).

#### Disassociation of LPS

The structural perturbation of LPS upon interaction with Nano-BA_P85_ was further detected by dynamic light scattering. LPS alone produced aggregates with a diameter centred at 7000 nm (Fig. 6d). The dramatic shift of the average size of LPS towards a lower value (≈ 2000 nm) was observed in the presence of Nano-BA_P85_, and the aggregation centred at 7000 nm totally disappeared (Fig. 6e). The appearance of a peak around 100 nm could correspond to the Nano-BA_P85_.

### Fluidity properties of the cell wall/membranes

Interactions of Nano-BAs with bacterial wall/membrane were evaluated in a fluorescence polarization study using DPH as a probe. DPH is a hydrophobic fluorescence compound that spontaneously incorporates in the hydrocarbon regions of lipid membranes. The transfer of DPH from the aqueous environment into the cell membranes results in a drastic increase in the intensity of the fluorescence emission of this probe. Furthermore, once the probe is incorporated into the lipid membrane, its fluorescence polarization is strongly dependent on the microenvironment. This provides valuable information concerning the membrane structure, specifically membrane microviscosity. We examined the time-dependent changes in the fluorescence polarization of DPH in *E. coli* and *S. aureus* cells following exposure to the tested formulations (Nano-BA_P85_, Nano-BA_PLGA_ and Pluronic^®^ P85 unimers). As shown in Fig. 7a, for *S. aureus* cells, there was a rapid decrease in the membrane microviscosity following the addition of Nano-BA_P85_ to the cell suspension. After 20 min of exposure to Nano-BA_P85_, the microviscosity levelled off and then remained constant throughout the duration of the experiment. Nano-BA_PLGA_ could also induce a similar decrease in the membrane microviscosity but to a reduced degree compared with Nano-BA_P85_. Pluronic^®^ P85 unimers exhibited a slight effect on the membrane microviscosity of *S. aureus* cells. A similar result was obtained for Nano-BA_P85_ and Nano-BA_PLGA_ for the membrane microviscosity of *E. coli* cells. Furthermore, Pluronic^®^ P85 unimers showed a moderate effect on the membrane microviscosity of *E. coli* cells, as observed by a steady decline in fluorescence.

**Fig. 7:** The effects of Nano-BA_P85_, Nano-BA_PLGA_ and Pluronic^®^ P85 unimers on the microviscosity of *E. coli* cells (**a**) and *S. aureus* cells (**b**). Significance: *p < 0.05, **p < 0.01, ***p < 0.001, significance represents Nano-BA_P85_ vs. Nano-BA_PLGA_ and Pluronic^®^ P85 unimers

### Assessment of the effect of Nano-BA_P85_ on the cytoplasmic membrane

#### Lipid membrane permeabilization

The ability of Nano-BA_P85_ to permeabilize artificial lipid membranes was investigated, ensuring the marked effect of Nano-BA_P85_ on membrane properties. This phenomenon was examined using liposomes mimicking the lipid composition of *E. coli* membranes (PG/CL/PE) and *S. aureus* membranes (PG/CL) [37]. Calcein was entrapped within these vesicles at a self-quenching concentration. An increase in its fluorescence reflected its dequenching due to membrane permeabilization and release of the dye. The kinetics of membrane disruption by the Nano-BA_P85_ was measured by monitoring the increases in fluorescence over time. As shown in Fig. 8a, entrapped calcein rapidly leaked from PE/CL/PG SUVs in a time-dependent manner upon exposure to Nano-BA_P85_. Nano-BA_P85_ could induce 93% leakage from PE/CL/PG SUVs and resulted in nearly complete leakage of calcein, which reached a value similar to that obtained with Polymyxin B (95%). Upon addition of the membrane-disrupting agent Triton X-100, an additional 5–7% increase in calcein leakage from the liposomes was observed and resulted in complete loss of calcein. The Nano-BA_PLGA_ also effectively caused the PE/CL/PG liposomes to leak calcein, but to a reduced degree compared with Nano-BA_P85_, with only 71% leakage observed during the incubation time. For PG/CL SUVs (Fig. 8b), greater release of calcein was induced by Nano-BA_P85_ (97%) than with Nano-BA_PLGA_ (76%). These results suggested that Nano-BA_P85_ could induce lipid membrane permeabilization at its MIC in artificial membranes representing the inner leaflet of *E. coli* or *S. aureus* membranes.

**Fig. 8:** Nano-BA_P85_-induced calcein release as a function of time. Nano-BA_P85_ were added to PG/CL/PE SUVs (**a**) and PG/CL SUVs (**b**) encapsulated with calcein. Cytoplasmic membrane potential variation of *E. coli* (**c**) and *S. aureus* (**d**) treated with Nano-BA_P85_ at 1 × MIC, as assessed by the release of the membrane potential-sensitive dye disC_3_-5. The fluorescence intensity was monitored at λ_ex_ = 622 nm and λ_em_ = 670 nm as a function of time. Effect of Nano-BA_P85_ on the cytoplasmic membrane permeability of *E. coli* cells (**e**) and *S. aureus* cells (**f**). The graphs were derived from average values of three independent trials

#### Membrane depolarization

The ability of Nano-BA_P85_ to depolarize the cytoplasmic membrane of *E. coli* and *S. aureus* cells was determined using the membrane potential-sensitive dye diSC_3-_5. Under the influence of a membrane potential, the dye can concentrate in the cytoplasmic membrane, resulting in self-quenching of fluorescence. Upon permeabilization and disruption of the cytoplasmic membrane, the membrane potential will dissipate and the diSC_3-_5 will release into the medium, causing a consequent increase in fluorescence intensity. As shown in Fig. 8c, the fluorescence intensity of disC_3_-5 was strongly quenched due to the dye that accumulated in the membrane. After the signal was stable for 5 min, Nano-BA_P85_ and Nano-BA_PLGA_ were added at various concentrations. When membrane depolarization was measured after addition of Nano-BA_P85_, we found a rapid increase in fluorescence intensity due to the collapse of the ion gradients that generated the membrane potential. Furthermore, Nano-BA_P85_ showed a similar depolarization capacity in *E. coli* and *S. aureus* cells, suggesting that Nano-BA_P85_ was effective against cytoplasmic membranes of both Gram-negative and Gram-positive bacteria. Comparatively, Nano-BA_PLGA_ showed a weaker membrane depolarization capability compared with Nano-BA_P85_. Taken together, Nano-BA_P85_ clearly induced *E. coli* and *S. aureus* membrane depolarization.

#### Cytoplasmic membrane permeability

We also determined the ability of Nano-BA_P85_ to permeabilize the cytoplasmic membrane of *E. coli* and *S. aureus* cells by measuring the release of cytoplasmic β-galactosidase with ONPG as the substrate. If Nano-BA_P85_ induced the permeabilization of the cytoplasmic membrane, ONPG could enter the cytoplasm and be degraded by β-galactosidase to produce o-nitrophenol, which was measured at an absorbance of 420 nm. As shown in Fig. 8e, f, Nano-BA_P85_ induced rapid increases in the absorption at 420 nm for both *E. coli* and *S. aureus* cells at 1 × MIC, which was similar to the results obtained for the positive control, in which the bacteria were lysed with 70% (v/v) isopropyl alcohol. In addition, there was no significant difference in cytoplasmic membrane permeabilization of Nano-BA_P85_ between the two types of bacterial cells.

#### In vivo anti-infective activity of Nano-BA_P85_

To evaluate the in vivo anti-infective activity and toxicity level of Nano-BA_P85_, *S. aureus* and/or *E. coli* was introduced into male KM mice intraperitoneally via a minimum lethal dose of 10^9^ CFU/mL (0.2 mL), which was first determined from the survival rate of mice at 48 h. At the lethal dose, 100% of mice died within 48 h post-injection. For both *S. aureus* and *E. coli*-infected mice (Fig. 9), Nano-BA_P85_ resulted in a significant drop in bacterial counts in ascites during the course of the treatments, which was more obvious than in the negative control group. The survival rate of the mice was observed for 7 days (Fig. 10). For *S. aureus* infection (Fig. 10a), treatment with Nano-BA_P85_ and Nano-BA_PLGA_ significantly prolonged the mean time until death compared with the untreated animals and BA group. Nano-BA_P85_ resulted in a significant reduction in the death rate after the treatments compared with Nano-BA_PLGA_. For *E. coli* infection (Fig. 10b), treatment with Nano-BA_PLGA_ and Nano-BA_P85_ also prolonged the mean time until death compared with the untreated animals and polymyxin B. For the mixed infection (Fig. 10c), all the mice died, except the mice in the Nano-BA_P85_ group, which had a survival rate of 100%, correlating well with the in vitro results.

**Fig. 9:** Colony formation units of bacteria in ascites of mice without any treatment (the negative control group) or treated with Nano-BA_P85_ for various periods of time

**Fig. 10:** Survival rates of mice intraperitoneally injected with *S. aureus* (**a**), *E. coli* (**b**) and mixed *S. aureus* and *E. coli* bacteria (**c**). Animals in each bacterial infection model group (n = 24) were randomly divided into four groups (n = 6, three female mice and three male mice) and then intraperitoneally injected with 200 μL of saline, BA solution, polymyxin B, Nano-BA_PLGA_ or Nano-BA_P85_ at doses of 100 mg/kg, 100 mg/kg, 30 mg/kg, 30 mg/kg and 30 mg/kg twice a day for 3 days. Data are expressed as the mean ± standard deviation based on the values obtained from the six mice in each group

## Discussion

In our preliminary study, PLGA-modified bacitracin A (Nano-BA_PLGA_) failed to manifest the desirable antibacterial potency due to limited solubility with longer PLGA blocks. In the search for new copolymers, the group of Pluronics has attracted significant attention from experimental medicine and pharmaceutical sciences during the last decade. Pluronic-modified bacitracin A self-assembled into micelles with a hydrophobic core composed of PPO segments and a hydrophilic shell composed of mixed PEO and bacitracin A segments. The antibacterial activity assay revealed the comprehensive result that all Pluronic-based Nano-BAs were more effective than Nano-BA_PLGA_ against both Gram-positive and Gram-negative bacteria. Thus, the addition of Pluronic copolymer (Pluronic^®^ F127, Pluronic^®^ P85 and Pluronic^®^ P123) did not merely provide a hydrophobic block to self-assemble micelles, but it also endowed the resulting Nano-BAs with desirable antibacterial efficiencies. Moreover, it is worth noting that Nano-BA_P85_ demonstrated the strongest antibacterial activities among the newly designed Nano-BAs, although the molecular weight of the hydrophobic block PPO (≈ 3 kDa) was much lower than that of Pluronic^®^ P123 (≈ 8 kDa). This result was different from our previous study indicating that the molecular weight of the hydrophobic block is correlated with the antibacterial potency [13]. Previous studies have demonstrated that Pluronic^®^ P85 can interfere with the membrane microviscosity of animal cells [38]. The hydrophobic PPO chains of Pluronic^®^ P85 unimers were immersed into the hydrophobic areas of the biomembrane, resulting in alterations of the membrane structure. Alterations in the physical state of membrane lipids can influence a number of important protein-mediated processes, including the transport of various ions and nutrients as well as membrane-bound enzymatic activities [39, 40]. However, there have been limited reports concerning the interaction between Pluronic^®^ P85 and the bacterial cell membrane. Thus, further studies are warranted to elucidate the antibacterial mechanism of Nano-BA_P85_ and the role played by Pluronic^®^ P85 in the antibacterial process.

Surface tension measurements indicated that Nano-BA_P85_ was much more tensioactive than Nano-BA_PLGA_, which was usually translated into a good membranolytic effect. Direct visual observation by TEM confirmed that the Nano-BA_P85_ induced significant rupture of the cell wall/membrane of both *S. aureus* and *E. coli* cells. For *S. aureus* cells, Nano-BA_P85_ could decrease the PG content in a concentration-and time-dependent manner. Bacitracin A has been shown to strongly inhibit Gram-positive bacteria by disturbing cell wall synthesis. The formation of Nano-BA_P85_ is expected to increase the local density of the BA mass on the surface, which could efficiently translate into excellent antibacterial activity. Lipopolysaccharide (LPS) is thought to be the major structural component of the outer membrane of Gram-negative bacteria and forms a protective wall to resist a variety of host defence molecules [34]. Therefore, we also investigated the role of LPS in bacterial susceptibility to Nano-BA_P85_. Surface pressure measurements indicated that Nano-BA_P85_ could cross the LPS monolayer even at an initial surface pressure of 35 mN/m, suggesting excellent LPS membrane permeability. The enhanced LPS monolayer permeability of Nano-BA_P85_ might result from the high binding affinity and insertion ability of Pluronic^®^ P85 with the hydrophobic lipid A domain of LPS. Hydrophobic PPO blocks could interact with LPS and as a synthetic carrier, facilitating the endocytosis of Nano-BA_P85_. In addition, Nano-BA_P85_ also showed strong LPS neutralization potency and could consequently dissociate the aggregated state of LPS, leading to a significant perturbation of the LPS packing organization.

The compromised cell wall/outer membrane may allow an increased influx of Nano-BA_P85_ into the periplasmic space. A large amount of Nano-BA_P85_ could cause sufficient permeabilization of the cytoplasmic membrane of both *S. aureus* and *E. coli* cells that allowed the passage of small molecules, such as ONPG, suggesting that a sequence of steps occurred at the membrane, beginning with depolarization (small ion permeability) and followed by more significant membrane disruption. Similar results were also observed in membranes mimicking liposomes. The calcein leakage assay monitored through fluorescence is well documented as a technique for probing antibacterial drug activity [41, 42]. Calcein is a relatively large, water-soluble molecule, and its release from liposomes is assumed to involve the formation of some type of pore in liposomes [43]. Nano-BA_P85_ could induce dye leakage from both PG/CL (representing the cytoplasmic membrane of *S. aureus*) and PG/CL/PE (representing the cytoplasmic membrane of *E. coli*), indicating a significant perturbation of membrane mimetics, and the slope of the time course of Nano-BA_P85_ was much higher than that of Nano-BA_PLGA_. Two phenomena may be responsible for the enhanced cytoplasmic damage potency of Nano-BA_P85_ compared with Nano-BA_PLGA_. (1) Higher local density of BA mass on the surface–The aggregation number of Nano-BA_P85_ (≈ 79) was much higher than that of Nano-BA_PLGA_ (≈ 47), suggesting a higher local density of BA mass on the surface. Since BA could disintegrate the bacterial cytoplasmic membrane of Gram-positive bacteria, massive BA on the surface could result in strong membrane permeabilization and cytoplasmic leakage. (2) Stronger membrane microviscosity-altering ability–This phenomenon might be attributed to the hydrophobic PPO chains of the Pluronic^®^ P85 unimers immersed in the hydrophobic areas of the biomembranes, resulting in alterations of the membrane structure and decreases in microviscosity (“membrane fluidization”). In addition, the uptake of Nano-BA_P85_ via the cell membrane may cause steric hindrance, leading to destruction of the organism by the formation of transient pores or channels and thus impairing the cellular machinery [44]. Taken together, Nano-BA_P85_ could first destroy the PG cell wall or bind predominantly to LPS, facilitating its entrance into the periplasmic space of bacterial cells. Then, further destabilization of the membrane based on the sinking raft model could result in cell death [45].

The in vivo experiments indicated that Nano-BA_P85_ was effective against bacterial peritonitis infection by *S. aureus* and *E. coli* alone or together in KM mice model, as evidenced by the high bacterial suppression and survival rate. In the future study, we will further determine the toxicity of Nano-BA_P85_ to major organs such as the liver and kidney. Usually, antibiotics are generally administered via oral or intravenous routes in order to treat infections, often resulting in undesired systemic side effects by nonspecific drug distribution in many different tissues and organs. Therefore, targeted delivery of antimicrobial drug to the infection site using nanoantibiotics is an exciting prospect in treating infectious diseases [46, 47]. Nano-BA_P85_ might target to the inflammatory tissue due to the enhanced permeability and retention (EPR) effect of inflammation, yielding not only better antibacterial effect but also lower systemic toxicity [48–53]. We will also analyse the antibacterial activity of Nano-BA_P85_ against the clinic isolated strains especially for the resistant strains.

## Conclusions

We have successfully developed Pluronic-based nano-self assemblies of bacitracin A with enhanced solubility and antibacterial activity for efficient in vivo therapeutic effects against bacterial peritonitis. The Pluronic-based Nano-BAs demonstrated a new membrane-targeting mechanism of action, which was different from its unassembled counterpart of bacitracin A. Compared with the other tested Nano-BAs, Nano-BA_P85_ was more efficient against bacteria both in vitro and in vivo, without causing significant toxicity to major organs. Currently, the field of nanoantibiotics is barely in its infancy in comparison to targeted nanomedicine for cancer and cardiovascular disease treatment, and there are very little data on the clinical applications, toxicity and antibacterial mechanisms of nanoantibiotics. In the present study, all the presented data will aid in the design of self-assembled nano-polypeptide antibiotic candidates for future therapeutic purposes with a clear antibacterial mechanism, and Nano-BA_P85_ could be a potential anti-infective agent for the treatment of bacterial peritonitis.

## Additional file

**Additional file 1.** Synthesis and Characterization of BA-PEO-PPO-PEO-BA
